The article "SeqBench: Integrated solution for the management and analysis of exome sequencing data" was published in 2014. Journal: BMC Res Notes.

# SeqBench: Integrated solution for the management and analysis of exome sequencing data

**DOI:** 10.1186/1756-0500-7-43

**Published:** 2014-01-20

**Authors:** Andreas Dander, Stephan Pabinger, Michael Sperk, Maria Fischer, Gernot Stocker, Zlatko Trajanoski

**Affiliations:** 1 Division for Bioinformatics, Biocenter, Innsbruck Medical University, Innsbruck, Austria; 2 Oncotyrol, Center for Personalized Cancer Medicine, Innsbruck, Austria; 3 AIT - Austrian Institute of Technology, Health & Environment Department, Molecular Diagnostics, Vienna, Austria; 4 ADSI, Austrian Drug Screening Institute, Innsbruck, Austria

**Keywords:** Sequencing, Exome, Data analysis, Web application, Cloud, Virtual machine image, Open-source

## Abstract

**Background:**

The rapid development of next generation sequencing technologies, including the recently introduced benchtop sequencers, made sequencing affordable for smaller research institutions. A widely applied method to identify causing mutations of diseases is exome sequencing, which proved to be cost-effective and time-saving.

**Findings:**

SeqBench, a web-based application, combines management and analysis of exome sequencing data into one solution. It provides a user friendly data acquisition module to facilitate comprehensive and intuitive data handling. SeqBench provides direct access to the analysis pipeline SIMPLEX, which can be configured to run locally, on a cluster, or in the cloud. Identified genomic variants are presented along with several functional annotations and can be interpreted in a family context.

**Conclusions:**

The web-based application SeqBench supports the management and analysis of exome sequencing data, is open-source and available at http://www.icbi.at/SeqBench.

## Findings

### Background

The introduction of next-generation sequencing (NGS) technologies has sparked a major revolution in biomedical research. Modern benchtop sequencers - such as the MiSeq (Illumina), PGM (life technologies), and 454 GS Junior (Roche) - generate only modest set-up and maintenance costs, and as a consequence genomic sequencing data are now produced at an unprecedented rate. At the same time, they are confronted with enormous challenges in data management, computer hardware requirements, and data analysis.

Exome sequencing is a widely used approach to elucidate the causing mutations of various diseases, including Mendelian disorders and cancer [1-3]. A plethora of tools for analyzing exome sequencing data are available, making efficient and standardized data analysis challenging for inexperienced users [4].

SIMPLEX [5] is a cloud-enabled analysis pipeline, which autonomously performs the complete workflow of exome sequencing data analysis. The pipeline is able to perform the following steps: (a) initial quality control, (b) intelligent data filtering and pre-processing, (c) sequence alignment to a reference genome, (d) SNP and INDEL detection, (e) functional annotation of variants, and (f) detailed report generation during various stages of the workflow.

SIMPLEX combines several established analysis applications (such as BWA and GATK) with in-house developed analysis tools (e.g. the quality report) into a tailored pipeline. Underlying applications can be configured using a variety of exposed parameters. The pipeline annotates identified variants using GATK, ANNOVAR, and SnpEff as well as a variety of attributes derived from the databases RefSeq, GO, KEGG, dbSNP, and the 1000 genomes project. Additionally, annotation scores from SIFT, PolyPhen2, PhyloP, MutationTaster, and LRT are added to the variants.

Recently, several software suites for handling exome sequencing data have been published, which differ in their provided feature set [6-9].

However, to the best of our knowledge there is currently no tool available which supports cloud computing and combines data management, data analysis, and result visualization into a single solution. Such an integrated solution would be of great help for labs without dedicated computational infrastructure. Additionally, the system should be easy to install and therefore be provided as a virtual machine (VM) image.

The new web-based application SeqBench embeds the established analysis pipeline SIMPLEX and provides a data acquisition module supporting data derived from Illumina and SOLiD platforms. This module guides the user through all stages of data entry. In addition, SeqBench provides a module to monitor ongoing SIMPLEX analyses and offers an intuitive interface to interpret computed results.

The preconfigured out of the box solution is very easy to install and presents itself as the ideal solution for inexperienced users. Yet, as SeqBench is completely open-source, it can be adapted and modified by experienced users to answer specific biological questions. Furthermore, SeqBench offers multiple customization options and can be configured to run the computationally expensive data analysis pipeline either in the cloud, on a high-performance computing infrastructure, or on a powerful local desktop machine using the provided VM image.

### SeqBench

SeqBench is organized in different modules as depicted in Figure 1. After logging in, a dashboard shows currently running SIMPLEX processes, results of finished analyses, and a list of available projects. New and existing projects can be added and modified using an intuitive data acquisition wizard. Users are guided through all necessary steps, making sure that project information and complementary data is entered in a consistent and coherent way. SeqBench allows users to upload and analyze raw sequencing data in FASTQ (Illumina) or CSFASTA/QUAL (SOLiD) format. As the analysis pipeline offers a wide variety of parameters to tailor the analysis to a specific biological problem, SeqBench offers a flexible system to set those parameters.

**Figure 1:** **Modules of SeqBench.** SeqBench is organized into the following modules: (i) data acquisition wizard for consistent data entry, (ii) dashboard displaying projects and analyses for the signed in user, (iii) connection to the analysis pipeline SIMPLEX, (iv) visualization of the data analysis results. The analysis pipeline SIMPLEX can run locally, on a cluster, or in the cloud. The system is secured by an authorization and authentication system (AAS), which uses as backend either a XML file or a dedicated web application.

A well chosen set of standard values is based on the suggestions by the used applications of SIMPLEX. SeqBench passes the uploaded raw files and selected parameter values on to SIMPLEX thus starting the analysis process. As output of the pipeline, files for several steps are created, SeqBench constantly monitors those output files and displays the progress in the result view. At the end of a pipeline run a summary of result files is generated, whereby selected files can be directly accessed via SeqBench.

The result visualization module in SeqBench allows users to access and download all generated analysis files. Furthermore, a table of identified SNPs and INDELs is displayed, including several functional annotations with outgoing links. Furthermore, all annotations found by SIMPLEX can be displayed as columns of this table. This table features dynamic column selection, real-time filtering, and sorting of mutations. Descriptive statistics about the filtered variants are illustrated in charts as depicted in Figure 2, which are updated dynamically after filtering. As SIMPLEX supports the analysis of multiple samples at once, SeqBench provides a combined view of identified variants to interpret results in their family context. Therefore, after uploading all files into SeqBench, one SIMPLEX analysis run can be started including all samples. Next, identified variants can be loaded into the variant table view, where they can be filtered and investigated in a combined way.

**Figure 2:** **Screenshot of SeqBench.** The presented result view shows applied location filtering, sorting, and dynamic column selection options. Pie charts display statistics about identified and filtered variants.

Access to the system is secured by an authorization and authentication system (AAS), which can be configured to use either a simple XML file or a web-based application for the usermanagement [10]. The AAS allows the assignment of different user roles with dedicated data access permissions, which are enforced within SeqBench.

SeqBench is open-source and distributed as a VM image that ships with a preconfigured AAS and a fully configured SIMPLEX pipeline. A detailed user manual provides information about installation, configuration, and usage of SeqBench as well as the installation process using VirtualBox as the virtual machine software which runs on Windows, Linux and Mac OS X ( https://seqbench.i-med.ac.at/SeqBench/doc/userManual.jsf). Details about how to use SIMPLEX in the cloud is provided in the SIMPLEX user manual ( http://icbi.at/software/simplex/simplex.shtml).

### Implementation

SeqBench is a Java EE 6 based web application running on a JBoss application server. It uses a relational database (PostgreSQL) accessed via an object relational mapper (Hibernate). JBoss Seam in combination with "Contexts and Dependency Injection" (CDI) is used as underlying framework. The presentation layer is based on Java Server Faces (JSF) and the JBoss Richfaces component library, which supports internationalization and input validation.

### Conclusion

SeqBench combines data management, data analysis, and result visualization into a single web-based platform. The complete software suite is distributed as a VM image providing several benefits to users such as easy installation, replication of analyses, or taking snapshots for archiving results (see recently published review [11]). To the best of our knowledge it is the only integrated solution that provides, amongst other features, SOLiD as well as cloud support.

SeqBench provides an intuitive user interface and facilitates comprehensive data acquisition through a wizard system and can be easily installed as an out of the box solution. The application covers the complete workflow from data acquisition to result interpretation and supports Illumina as well as SOLiD data. In conclusion, SeqBench is a light-weight and effective solution for the streamlined integration of data management and analyses of exome sequencing data.

## Availability and requirements

• **Project name:** SeqBench

• **Project home page:**http://www.icbi.at/SeqBench

• **SVN access:**http://www.icbi.at/svnseqbench/seqbench/trunk

• **Operating system:** Platform independent

• **Programming language:** Java

• **Other requirements:** VirtualBox

• **License:** GNU AGPL

• **Any restrictions to use by non-academics:** no

## Abbreviations

AAS: Authorization and Authentication System; AGPL: Affero General Public License; NGS: Next-Generation Sequencing; GO: Gene ontology; KEGG: Kyoto Encyclopedia of Genes and Genomes; VM: Virtual machine.

## Competing interests

The authors declare that they have no competing interests.

## Authors contributions

AD, SP, MS, and MF developed SeqBench. AD designed the database scheme. SP and GS implemented the front-end of the application. MS developed the results report view. MF integrated SIMPLEX into SeqBench. GS and ZT conceived the project and suppervised the development. All authors participated in debugging and testing of SeqBench, and assisted in preparation of the article. All authors read and approved the final manuscript.
